The article "Correlation Analysis and Application of Respiratory and Lung Diseases in Pediatrics of Traditional Chinese Medicine Based on Factor Analysis Method" was published in 2022. Journal: Comput Math Methods Med.

# Correlation Analysis and Application of Respiratory and Lung Diseases in Pediatrics of Traditional Chinese Medicine Based on Factor Analysis Method

**DOI:** 10.1155/2022/4550039

**Published:** 2022-08-31

**Authors:** Shengnan Sun, Lingling Zhuang, Ming Cao

**Affiliations:** Traditional Chinese Medicine Academy of Science of Jilin Province, Changchun Jilin 130021, China

## Abstract

Many scholars have studied the influencing factors of children's lung infection, whether it is the region or the environment, or the living air quality of the mother during pregnancy. Western medicine is the most frequently used medicine, but Chinese medicine has more remarkable characteristics in treating children's lung diseases. For viral invasive diseases, people often use antibiotics to treat them. Children's lung conditions are too fragile, and taking antibiotics will lead to the damage of *Staphylococcus* in the lungs, resulting in pulmonary respiratory insufficiency. Although the conditioning time of traditional Chinese medicine is longer than that of western medicine, traditional Chinese medicine will not cause secondary damage to the lungs. In this paper, we introduce factor analysis and principal component analysis and compare the performance of the three analysis methods by using data such as cure rate, improvement rate, mortality rate, and drug taking frequency as evaluation indexes. In the model comparison, the accuracy rate of factor analysis method is over 97%, while the error rate is below 5%. Compared with the other two analysis methods, this method has a better application effect. Finally, we compare the comprehensive scores of eigenvalues of the three analysis methods. From 2016 to 2021, the comprehensive scores of factor analysis gradually increased.

## 1. Introduction

Children's lungs are easily infected by viruses, and circulating diseases such as pneumonia have great influence on children's lungs, which may cause irreversible damage [1]. By analyzing the blood gas performance of children, we can get some children's lung diseases related to clinical analysis, and the study can find different clinical manifestations and injury degrees of children [2]. Children's lung disease is one of the most common and complicated diseases in pediatric medicine. Before the Soviet Union was decomposed, good achievements were made in the treatment and effective control of children's lung disease [3]. The question why children's lungs are most susceptible to diseases has also attracted the attention of many researchers. Is it related to geography and environment? We statistically analyzed the number of children infected with lung diseases in various regions and found that geographical environment is one of the important pathological reasons [4]. Generally, we can take antibiotics to treat viral infections. However, studies have found that in children's lung diseases, taking antibiotics will lead to the damage of *Staphylococcus* in children's lungs, which will lead to pulmonary respiratory insufficiency [5]. The complication principle of children's lung diseases may lie in the air quality of mothers during lactation. We should pollute the living air quality of pregnant women, which is beneficial to the development of children's lungs [6, 7]. MRI findings of pneumonia caused by mycoplasma pneumoniae, *Streptococcus pneumoniae*, and other pathogens in children and abnormalities of lung parenchyma, pleura, and lymph nodes have good features on MRI. Contrast enhancement may be useful in distinguishing active inflammatory and noninflammatory changes, and MRI is especially useful in the follow-up of chronic lung diseases in children [8, 9]. Comparing the pathological conditions of two children, it is particularly difficult to determine the causes of these lesions and distinguish tumor process from infection. Patients with intrathoracic myopathy should be considered in the differential diagnosis of pulmonary and mediastinal mass lesions [10]. The parameters of traditional factor model are different among regulator variables, so a semiparametric moderation factor modeling method is proposed, which is feasible in parameter recovery and ability to distinguish different measurement invariance models [11]. This paper selects the relevant financial data of 10 listed real estate companies, such as Xiangjiang Holdings, Yunnan Chengtou, and Wantong Real Estate, evaluates their financial indicators and nonfinancial indicators by factor analysis, and makes quantitative and qualitative analysis [12–14]. The incidence and spread speed of the Novel Coronavirus are predicted and classified by machine learning algorithms [15]. It is very important to analyze the soil quality factors and quantitatively evaluate the soil quality in karst rocky desertification areas for providing the living conditions [16]. In selecting excellent genes of plants, the relationship between complex factors and variables can also be studied by factor analysis, and finally, seeds with good fruit quality can be selected [17–20]. Using different ultraviolet spectra, factor analysis was adopted to measure some antibacterial drugs [21]. The correlation among carcass was used as false phenotypes in genetic evaluation, and principal component method and variable rotation algorithm were used to extract factors [22]. In enterprise application, exploratory and confirmatory factor analysis is used to verify employees' self-leadership ability [23, 24]. This method studies the factors of the formation of dandruff in adolescents and uses principal component analysis to find out the main factors affecting dandruff in normal people [25].

The article "Correlation Analysis and Application of Respiratory and Lung Diseases in Pediatrics of Traditional Chinese Medicine Based on Factor Analysis Method" was published in 2022. Journal: Comput Math Methods Med.

## 2. Development Trend of Traditional Chinese Medicine

### 2.1. Development of Chinese Medicine Abroad

Chinese medicine has spread abroad for more than 2,000 years. As early as Qin and Han Dynasties, Chinese medicine spread to Japan, Korea, Vietnam, and other neighboring countries. Subsequently, the medical exchanges between Southeast Asian countries and China continued to deepen, and traditional Chinese medicine began to spread widely in Arab countries. Later, infectious diseases such as smallpox broke out, which made vaccination spread to five continents and four oceans. Once, the president of the United States also told his own experience of receiving acupuncture treatment after the operation of broad tail inflammation in China, which made acupuncture spread quickly throughout the United States and western countries. Chinese acupuncture has become a major treatment measure for medical health in the world. Nowadays, Chinese medicine has spread to more than 100 countries and regions in the world and has gradually become one of the important ways for people in the world to choose medical care.

### 2.2. Trends in Chinese Medicine Trade

The outbreak of COVID-19 pandemic in recent years has made the supply of drugs even more cramped. Studies have shown that Lianhua Qingpox Capsule has a protective effect on Novel Coronavirus, which makes the export of traditional Chinese medicine reach the peak in recent years. The average annual growth rate of Chinese medicine export has reached more than 10% in recent five years, and the number of Chinese medicines exporting countries has reached nearly 200 countries or regions. At the same time, some ready-for-use traditional Chinese medicine trademarks and brands with international influence have been formed, such as Compound Danshen Dropping Pills, Compound Banlangen, Huoxiang Zhengqi Liquid, Kanglaite Capsule, Kanglaite Injection, and Lianhua Qingpox Capsule. The total drug exports in China from 2016 to 2021 are shown in Figure 1.

## 3. Different Analysis Algorithms

### 3.1. Principal Component Analysis Algorithm

Principal components of the influence of traditional Chinese medicine on children's lungs are

(1) $$\begin{array}{c} F_{i}=a_{1}X_{1}+a_{2}X_{2}+\cdots +a_{i}X_{i}. \end{array}$$

Eigenvalues and eigenvectors of principal components of the influence of traditional Chinese medicine on children's lungs are

(2) $$\begin{array}{c} A={\left(a_{ij}\right)}_{p\times m}=\left(a_{1},a_{2}..,a_{m}\right),\\ {Ra}_{i}=\lambda_{i}a_{i}. \end{array}$$

The correlation of *λ*_*i*_ is *λ*_1_ ≥ *λ*_2_ ≥ ⋯≥*λ*_*p*_ ≥ 0, and *λ*_*i*_ is different from each other.

The article "Correlation Analysis and Application of Respiratory and Lung Diseases in Pediatrics of Traditional Chinese Medicine Based on Factor Analysis Method" was published in 2022. Journal: Comput Math Methods Med.

Calculate orthogonal matrices:

(3) $$\begin{array}{c} A^{\prime }A=I. \end{array}$$

Calculate the covariance:

(4) $$\begin{array}{c} \mathrm{cov}\left(F_{i},F_{j}\right)=\lambda_{i}\delta_{ij},\\ \delta_{ij}=\left\{\begin{array}{cc} 0 & i\neq j\\ 1 & i=j. \end{array}\right. \end{array}$$

Set the principal components of the influence of TCM on children's lungs as functions:

(5) $$\begin{array}{c} {\left(F_{1},F_{2},..,F_{m}\right)}^{\prime }=A^{\prime }X. \end{array}$$

Calculate the sum of squares of *X* coefficients in the principal components of TCM's influence on children's lungs:

(6) $$\begin{array}{c} \overset{p}{\underset{k=1}{\sum }}a_{ki}^{2}=1. \end{array}$$

Combine principal component functions:

(7) $$\begin{array}{c} F=\overset{m}{\underset{i=1}{\sum }}\left(\lambda_{i}/p\right)F_{i}. \end{array}$$

Firstly, it uses dimension reduction technology to replace the original multiple variables with a few comprehensive variables, which concentrate most of the information of the original variables. Secondly, it evaluates the objective economic phenomena scientifically by calculating the score of the comprehensive principal component function. Thirdly, it focuses on the comprehensive evaluation of information contribution and influence in application.

The analysis steps of principal component analysis are defined as follows:

Step 1: select initial variables

Step 2: choose whether to use covariance matrix or correlation matrix to find principal components according to the characteristics of initial variables

Step 3: calculate the eigenvalues and eigenvectors of the covariance matrix or correlation matrix

Step 4: determine the number of principal components

Step 5: the economic meaning of principal component is determined by several indexes with greater weight in each linear combination

### 3.2. Factor Analysis Algorithm

Variables of the influence of traditional Chinese medicine on children's lungs are as follows:

(8) $$\begin{array}{c} X_{j}=b_{j1}Y_{1}+b_{j2}Y_{2}+\cdots +b_{jm}Y_{m}+\epsilon_{j},\\ \mathrm{cov}\left(\epsilon_{j},Y_{i}\right)=0, \end{array}$$

where *ϵ*_*j*_ and *Y*_*i*_ represent special factors. The covariance between them is 0, and the formula is cov(*ϵ*_*j*_, *Y*_*i*_) = 0.

The variable factor load matrix is

(9) $$\begin{array}{c} B={\left(b_{ij}\right)}_{p\times m}=\hat{B}C,\\ \hat{B}=\left(\sqrt{\lambda_{1}}a_{1},\sqrt{\lambda_{2}}a_{2},\cdots ,\sqrt{\lambda_{m}}a_{m}\right). \end{array}$$

Its matrix relationship is

(10) $$\begin{array}{c} B^{\prime }B\neq I. \end{array}$$

The correlation of variables is

(11) $$\begin{array}{c} X_{i}Y_{j}=b_{ij}. \end{array}$$

Calculate the covariance:

(12) $$\begin{array}{c} \mathrm{cov}\left(Y_{i},Y_{j}\right)=\delta_{ij},\\ \delta_{ij}=\left\{\begin{array}{cc} 0 & i\neq j\\ 1 & i=j. \end{array}\right. \end{array}$$

The contribution value of factor *Y*_*i*_ to *X* is

(13) $$\begin{array}{c} v_{i}=\overset{p}{\underset{k=1}{\sum }}{b_{ki}}^{2}\left(\neq \lambda_{i}\right). \end{array}$$

The expression for calculating the score value of variable factor is

(14) $$\begin{array}{c} {\left(Y_{1},Y_{2},..,Y_{m}\right)}^{\prime }=B^{\prime }R^{-1}X. \end{array}$$

The factor similarity function is

(15) $$\begin{array}{c} \overset{m}{\underset{i=1}{\sum }}{b_{ij}}^{2}+{\sigma_{j}}^{2}={h_{j}}^{2}+{\sigma_{j}}^{2}=1, \end{array}$$

where *h*_*j*_^2^ stands for common degree and *σ*_*j*_^2^ stands for special variance. Commonality refers to the sum of squares of the loads of each variable in each common factor.

The article "Correlation Analysis and Application of Respiratory and Lung Diseases in Pediatrics of Traditional Chinese Medicine Based on Factor Analysis Method" was published in 2022. Journal: Comput Math Methods Med.

The factor covariance expression is

(16) $$\begin{array}{c} \mathrm{cov}\left(\epsilon_{i},\epsilon_{j}\right)=\delta_{ij}{\delta_{j}}^{2}. \end{array}$$

Synthesize the score function expression of each factor:

(17) $$\begin{array}{c} Y=\overset{m}{\underset{i=1}{\sum }}\left(v_{i}/p\right)Y_{i},\\ \frac{v_{i}}{p}=\frac{v_{i}}{v_{1}+v_{2}+\cdots +v_{m}}. \end{array}$$

The standardized formulas of various indicators of the influence of traditional Chinese medicine on children's lungs are as follows:

Inverse indicator:

(18) $$\begin{array}{c} {x_{i}}^{\prime }=1/x_{i} \end{array}$$

Moderate indicators:

(19) $$\begin{array}{c} {x_{i}}^{\prime }=1/\left(1+\left|a_{i}-x_{i}\right|\right) \end{array}$$

Therefore, the unified standardization of indicators is

(20) $$\begin{array}{c} Y_{ij}=\frac{x_{ij}-x_{i}}{s_{j}}. \end{array}$$

Test the index:

(21) $$\begin{array}{c} \frac{1}{N-1}\overset{N}{\underset{j-1}{\sum }}{x_{ij}}^{\prime }x_{ij},R=\left\{r_{ij}\right\}. \end{array}$$

The analysis steps of factor analysis is defined as follows:

Step 1: choose the variables for analysis

Step 2: calculate the correlation coefficient matrix of the selected original variables

Step 3: put forward common factors

Step 4: factor rotation

Step 5: calculate factor scores

Find out the factor score of each sample. If you have the factor score value, you can use these factors in many analyses, such as using the factor score as a variable in cluster analysis and a regression factor in regression analysis.

## 4. Experiment

### 4.1. Data Processing

Traditional Chinese medicine has the phenomenon of multiple names, abbreviations, and different places of origin, which has a great impact on the later statistics. Therefore, before formal analysis, we need to preprocess the data and unify the drug names, as shown in Table 1.

The article "Correlation Analysis and Application of Respiratory and Lung Diseases in Pediatrics of Traditional Chinese Medicine Based on Factor Analysis Method" was published in 2022. Journal: Comput Math Methods Med.

Standardize and unify the names of traditional Chinese medicines for treating lung diseases, and make a preliminary analysis of the frequency of medication. Select high-frequency drugs to test whether they meet the conditions of factor analysis. KMO test is carried out on lung traditional Chinese medicine with high-frequency medication. If the KMO value is greater than 0.6, it has a good linear relationship and is also suitable for factor analysis in Table 2.

The covariance is calculated by factor analysis, and the gravel diagram composed of each factor variable is shown in Figure 2.

It can be seen in Figure 2 that 72-75 factors are the most stable, that is, 72-75 factors are the most appropriate.

### 4.2. Model Comparison

There are many analytical methods for TCM treatment of children's lung diseases. In order to find the best analytical method, we compare the performance of various analytical methods on the cure rate, improvement rate, mortality rate, drug taking frequency, and other indicators of lung pediatrics.

The data analysis and statistics of pediatric lung diseases by factor analysis are shown in Table 3.

The application data of pulmonary pediatric treatment evaluation index are counted into a bar chart as shown in Figure 3.

The data analysis and statistics of pediatric lung diseases by ratio analysis method are shown in Table 4.

The application data of pulmonary pediatric treatment evaluation index are counted into a bar chart as shown in Figure 4.

The data analysis and statistics of pediatric lung diseases by trend analysis method are shown in Table 5.

The application data of pulmonary pediatric treatment evaluation index are counted into a bar chart as shown in Figure 5.

### 4.3. Contrast Experiment

By comparing the performance of three kinds of analysis methods, we can get the index data of children's lung treatment. Using the factor analysis method, we can get better statistical results. In order to further verify the best effect of this method, we use the factor analysis and other two analysis methods to compare the comprehensive scores of eigenvalues from 2016 to 2021, as shown in Figures 6–8.

Comprehensive evaluation refers to the method of using systematic and standardized methods to evaluate multiple indicators and units at the same time. The comprehensive score is the final index to measure the advantages and disadvantages of each evaluation object, and through ranking the comprehensive score, find out the best scheme.

The article "Correlation Analysis and Application of Respiratory and Lung Diseases in Pediatrics of Traditional Chinese Medicine Based on Factor Analysis Method" was published in 2022. Journal: Comput Math Methods Med.

## 5. Conclusion

Children's pathological conditions have always been a concern for parents. In recent years, western medicine treatment is still popular because of its quick effect and short time. However, people ignore that traditional Chinese medicine is a radical medicine for human body conditioning. Children's lung disease is a common kind of children's disease. We put forward factor analysis to analyze the correlation of pediatric respiratory lung disease in traditional Chinese medicine. The conclusions are as follows:

1. Factor analysis has good data analysis ability for complex pathological factors, and the data accuracy of traditional Chinese medicine for children's lung diseases is high
2. Comparing the performance of the three data analysis methods mentioned in this paper, the accuracy of factor analysis method reaches more than 90%, far exceeding the other two analysis methods
3. In the contrast experiment, the comprehensive score of the eigenvalues of the three analysis methods is carried out, and the comprehensive score of factor analysis method gradually increases, while the trend analysis method can only see one trend, which cannot reach a higher accuracy

## Figures and Tables

**Figure 1:** Total exports of traditional Chinese medicine in China from 2016 to 2021.

**Figure 2:** Lithotripsy diagram of medication frequency factor of lung diseases.

**Figure 3:** Performance comparison of evaluation indexes of children's lung treatment.

**Figure 4:** Performance comparison of evaluation indexes of children's lung treatment.

**Figure 5:** Performance comparison of evaluation indexes of children's lung treatment.

**Figure 6:** Comprehensive scores of factor analysis in recent years.

**Figure 7:** Comprehensive scores of ratio analysis in recent years.

**Figure 8:** Comprehensive scores of trend analysis in recent years.

**Table 1:** Standardization and unification of Chinese medicine names.

Drug serial number	Before specification	After specification
1	Panax notoginseng powder	Panax notoginseng
2	Yunling	Poria cocos
3	Polygonatum sibiricum	Polygonatum sibiricum
4	Patchouli	Agastache rugosa
5	Rhizoma Rehmanniae	Rehmannia glutinosa
6	Whole insect	Scorpion
7	Dismiss Rhizoma Atractylodis	Atractylodes lancea
8	Grass nut	Tsaoko
9	Grass river cart	Paris polyphylla
10	Xiaoyaozhu	Xu Changqing
11	White ginseng	Ginseng

**Table 2:** KMO test results.

Drug name	Degree of freedom	Significance
Poria cocos	4755	0
Xu Changqing	3782	0
Ginseng	4003	0
Atractylodes lancea	3431	0
Rehmannia glutinosa	2546	0

**Table 3:** Application data of factor analysis in pediatric treatment of lung.

Evaluation index	Accurate value	Error value	*F*1	Recall rate	ROC
Cure rate	97.89%	3.57%	78.56%	76.54%	80.54%
Rate of improvement	96.57%	4.21%	77.92%	75.83%	82.34%
Mortality rate	98.34%	4.45%	79.65%	75.52%	81.49%
Drug use rate	96.39%	3.86%	78.97%	78.48%	81.78%

The article "Correlation Analysis and Application of Respiratory and Lung Diseases in Pediatrics of Traditional Chinese Medicine Based on Factor Analysis Method" was published in 2022. Journal: Comput Math Methods Med.

**Table 4:** Application data of ratio analysis in pediatric treatment of lung.

Evaluation index	Accurate value	Error value	*F*1	Recall rate	ROC
Cure rate	73.45%	12.68%	56.55%	46.54%	60.54%
Rate of improvement	78.65%	13.21%	57.82%	45.88%	52.34%
Mortality rate	72.76%	12.25%	58.49%	47.54%	51.89%
Drug use rate	74.58%	14.51%	57.25%	52.48%	55.78%

**Table 5:** Application data of trend analysis method in pediatric treatment of lung.

Evaluation index	Accurate value	Error value	*F*1	Recall rate	ROC
Cure rate	53.47%	32.66%	39.55%	36.59%	40.44%
Rate of improvement	58.66%	33.25%	41.82%	37.67%	42.74%
Mortality rate	62.76%	32.28%	40.46%	40.04%	43.86%
Drug use rate	54.56%	34.54%	39.23%	38.58%	42.38%

## Data Availability

The experimental data used to support the findings of this study are available from the corresponding author upon request.
